# One-year outcome and survival analysis of deferred ventricular septal repair in cardiogenic shock supported with mechanical circulatory support

This article has been retracted.

**DOI:** 10.1371/journal.pone.0256377

**Published:** 2021-08-18

**Authors:** Jahanzeb Malik, Faizan Younus, Asmara Malik, Muhammad Umar Farooq, Ahmed Kamal, Muhammad Shoaib, Hesham Naeem, Ghazanfar Rana, Abdul Sattar Rana, Muhammad Usman, Shahid Khalil

**Affiliations:** 1 Department of Cardiology, Rawalpindi Institute of Cardiology, Rawal Road, Rawalpindi, Pakistan; 2 Department of Community Medicine, National University of Medical Sciences, Rawalpindi, Pakistan; 3 Department of Cardiology, Pakistan Institute of Medical Sciences, Islamabad, Pakistan; 4 Department of Cardiothoracic Surgery, Mega Medical Complex Hospital, Rawalpindi, Pakistan; 5 Department of Cardiology, St. Luke’s General Hospital, Kilkenny, Ireland; IRCCS Policlinico S.Donato, ITALY

## Abstract

**Background and objective:**

The effectiveness of deferred surgical repair of ventricular septal rupture (VSR) post-myocardial infarction (MI) with cardiogenic shock remains limited to case reports. Our study aimed to investigate the outcomes and survival analysis following mechanical circulatory support (MCS) in patients after VSR who develop cardiogenic shock.

**Methods:**

We analyzed 27 patients with post-MI VSR and cardiogenic shock who received deferred surgical repair while stabilized on MCS between January 2018 and March 2020. After normality test adjustments, continuous variables were expressed as mean ± standard deviation (SD). These were compared using the Mann-Whitney U test and Student’s t-test. Categorical variables were compared using chi-square or Fisher’s exact test. To identify predictors of operative mortality, univariate analysis of clinical characteristics and interventions followed by logistic regression was carried out. P-value of < 0.05 was considered significant.

**Results:**

All patients had preoperative MCS. Emergency repair was avoided in all the patients. The mean age of the participants was 64.96 with the majority being males (74.1%). On average, the mean time from MI to VSR repair was 18.85 days. Delayed revascularization was associated with increased mortality (OR 17.500, 95% CI 2.365–129.506, P = 0.005). Other factors associated with increased mortality were ejection fraction (EF), three-vessel disease, Killip class, early surgery, and prolonged use of inotropes. The operative mortality was 11% with an overall mortality of 33.3%. The one-year survival rate was 66.7%.

**Conclusion:**

The use of MCS in adjunct to a deferred surgical approach shows an improved survival outcome of patients with VSR complicated by cardiogenic shock. Further investigations are required regarding the optimal time for MCS and surgical repair.

## Introduction

Ventricular septal rupture (VSR) is a serious complication after an acute myocardial infarction (MI). The incidence of VSR was 1% to 3% in the era before accessible reperfusion practices [1]. However, the incidence has declined in recent years to around 0.3% following the emergence of thrombolysis and primary percutaneous coronary intervention (PPCI) [2]. SHOCK trial has shown that VSR typically develops 10 to 24 hours after acute MI and is not dependent upon the reperfusion strategy [3]. This finding was later validated by GUSTO-I and APEX-AMI trials [4, 5]. The prognosis is grave with a reported mortality of 23% to 80%(1). The mortality rate increases if cardiogenic shock develops before surgery [6]. In some studies, the delayed surgical approach yields better results as compared to emergency surgery [7, 8]. However, there is no agreement on the optimal time of surgery for VSR with cardiogenic shock.

Various studies report high mortality following an emergent surgical repair of VSR [9, 10]. However, the patient characteristics and results vary in studies related to delayed and emergent surgery. There is an increased use of mechanical support devices (MCS) in patients planned for emergency surgery as compared to the patients planned for delayed surgery. Hence, only hemodynamically stable patients usually undergo delayed surgery. This can be a factor in a better outcome for such patients. The impact of delayed surgery in patients with cardiogenic shock supported by MCS is only limited to case reports and there is a paucity of literature on this aspect [11].

This study aimed to investigate the post-operative and one-year survival of VSR repair in patients with cardiogenic shock who were put on MCS and deferred surgical repair.

## Methods

### Study design and patient selection

This study was approved by Mega Medical Complex (ID#MMC/07/18), and written, informed consent was waived off by the review board. A retrospective analysis was performed on 42 consecutive patients admitted with post-MI VSR at our institute between January 2018 and March 2020. Inclusion criteria were any patient admitted with acute MI and evidence of VSR who had emergency left heart catheterization or thrombolysis with alteplase followed by routine coronary angiography. Patients who died before VSR repair were included. Those not for MCS were excluded. After database search, 27 patients fulfilled the inclusion criteria. Of the 15 patients, 11 died before surgery and 7 of them had either intra-aortic balloon pump (IABP) or extracorporeal membrane oxygenation (ECMO).

Acute MI was diagnosed with typical chest pain and an elevation of serum troponin T > 14 ng/L with an electrocardiogram (EKG) evidence of > 2 mm ST-segment elevation in precordial leads or > 1 mm ST-elevation in the limb leads. A thorough chart review and analysis of the clinical profile was completed for medical and surgical units. Initial vital signs were used to determine the hemodynamics of each patient. VSR was defined as a defect in the septal myocardium visualized either on cardiac catheterization or echocardiogram. Cardiogenic shock was defined as systolic blood pressure of < 90 mmHg for > 30 min or use of inotropes and vasopressors to maintain a systolic blood pressure of > 90 mmHg, impaired organ perfusion presenting as altered mental status, cold peripheries, and oliguria.

### Echocardiography

All patients underwent an echocardiogram with verification of VSR by transthoracic (TTE) or trans-esophageal (TEE) echocardiography. This was done within an average of 2 hours and 46 minutes of admission. VSR was defined as a defect in the ventricular septum with significant left to right shunt on color Doppler. The VSR was identified as apical or basal on TTE and confirmed before surgical intervention by TEE. Ejection fraction (EF) was calculated by the modified Simpson’s method.

### Cardiac catheterization

After diagnosis of acute MI and/or VSR, all patients underwent a left heart catheterization with placement of IABP, ECMO, and/or left ventricular assist device (LVAD, Heartmate II, Abbott, USA.). Impella was not used in any of these patients as it is not available for reimbursement at our institute. Initiation of IABP with or without ECMO was done to maintain hemodynamic stability. Coronary artery disease (CAD) was defined as the involvement of one or more lesion stenosis of greater than 70% and left main stenosis of more than 50%. Lesions amenable to PPCI were addressed on index coronary angiogram with drug-eluting stents which was defined as early revascularization. Early revascularization was carried out in those patients who were not diagnosed with a VSR at presentation of acute MI. Delayed revascularization was defined as coronary artery bypass graft surgery (CABG) at the time of VSR repair.

### Outcomes

The primary outcome was all-cause mortality, defined as death from any cause after MCS with or without VSR repair and concomitant CABG. Additional outcomes included clinical characteristics, location of coronary artery disease, interventions, their complications, and use of MCS. Early VSR repair was defined as surgery within 7 days and delayed closure was defined as surgery after at least 10 days. Follow-up was done by telephonic interview to the patient or their attendants. All patient data is available within the (S1 File).

### Statistical analysis

Statistical analysis was done on the statistical package for social sciences (SPSS) version 26 (IBM, Armonk, NY). Continuous variables were summarized as mean ± standard deviation (SD). Depending on the normality of distribution, the Shapiro-Wilk test or Mann-Whitney U test was applied for comparing variables between the groups. Categorical variables were expressed as frequency and percentage. Comparison between survivors and non-survivors was performed by Student’s t-test, Fischer’s exact test, and Chi-square test for continuous and categorical variables respectively. To identify factors associated with mortality, univariate analysis of pre-and post-operative variables was performed. Logistic regression analysis was done for significant univariate risk factors. Survival function was presented as Kaplan-Meier survival curve and comparisons were performed with the log-rank test. A P-value of less than 0.05 was considered significant.

## Results

A total of 27 patients had delayed VSR repair on MCS who fulfilled our study criteria. The mean age was 64.96 ± 8.69 with the majority being males (74.1%) and having diabetes (63%). Two patients had a history of CAD. A coronary angiogram was done in all the patients. Non-survivors were more likely to have three-vessel disease (77.8% vs. 5.6%, P = 0.001), while survivors were more likely to have single-vessel disease (55%, P = 0.005). Left anterior descending artery (LAD) was the most common culprit lesion (66.7%) in both groups and anterior MI was the most common type of MI. Mean ejection fraction (EF) at admission was more in survivors (30.28 ± 7.16 vs. 19.44 ± 6.34, P = 0.118) with the apical septum being the most common type of VSR in both categories. Four out of nine patients did not survive with basal VSR while five out of eighteen patients died with apical VSR. Table 1 shows the demographic data and clinical characteristics in both groups.

**Table 1:** Demographic data and clinical characteristics.

	All (n = 27)	Survivors (n = 18)	Non-survivors (n = 9)	P-value
**Age in years (Mean ± SD)**	64.96 ± 8.69	65.72 ± 8.83	63.44 ± 8.66	0.200
**Males n(%)**	20 (74.1)	15 (83.3)	5 (55.6)	0.121
**Females n(%)**	7 (25.9)	3 (16.7)	4 (44.4)	0.175
**DM n(%)**	17 (63)	11 (61.1)	6 (66.7)	0.778
**HTN n(%)**	10 (37)	9 (50)	1 (11.1)	0.057
**Smoker n(%)**	9 (33.3)	4 (22.2)	5 (55.6)	0.083
**CKD n(%)**	3 (11.1)	2 (11.1)	1 (11.1)	1.0
**Dyslipidemia n(%)**	7 (25.9)	4 (22.2)	3 (33.3)	0.535
**BMI (Mean ± SD)**	30.22 ± 4.25	30.89 ± 4.48	28.89 ± 3.62	0.177
**EF (Mean ± SD)**	26.67 ± 8.54	30.28 ± 7.16	19.44 ± 6.34	0.118
**Type of MI n(%)**				
** Anterior**	18 (66.7)	13 (72.2)	5 (55.6)	0.391
** Inferior**	9 (33.3)	5 (27.8)	4 (44.4)	0.432
**Duration of MI**	38.89 ± 21.64	37.56 ± 21.89	41.56 ± 22.19	0.007
**Culprit vessel n(%)**				
** LAD**	18 (66.7)	13 (72.2)	5 (55.6)	0.391
** RCA**	9 (33.3)	5 (27.8)	4 (44.4)	0.432
**Single vessel n(%)**	10 (37)	10 (55.6)	0	0.005
**Two vessel n(%)**	9 (33.3)	7 (38.9)	2 (22.2)	0.667
**Three vessel n(%)**	8 (29.6)	1 (5.6)	7 (77.8)	0.001
**Type of VSR n(%)**				
** Apical**	18 (66.7)	13 (72.2)	5 (55.6)	0.391
** Basal**	9 (33.3)	5 (27.8)	4 (44.4)	0.432
**Anticoagulant n(%)**				
**UFH**	17 (63)	13 (72.2)	4 (44.4)	0.159
**Enoxaparin**	6 (22.2)	3 (16.7)	3 (33.3)	0.326
**Bivalirudin**	4 (14.8)	2 (11.1)	2 (22.2)	0.444
**Multi-organ dysfunction n(%)**	13 (48.1)	8 (44.4)	5 (55.6)	0.586
**MAP (Mean ± SD)**	88.04 ± 11.75	95.39 ± 5.81	73.33 ± 3.50	0.007
**HR/min (Mean ± SD)**	116.11 ± 27.05	98.78 ± 9.50	150.78 ± 12.56	0.043

Diabetes mellitus. (DM); Hypertension (HTN); Chronic kidney disease (CKD); Body mass index (BMI); Ejection fraction (EF); Myocardial infarction (MI); Left anterior descending artery (LAD); Right coronary artery (RCA); Ventricular septal rupture (VSR); Unfractionated heparin (UFH); Mean arterial pressure (MAP); Heart rate (HR).

All operations were performed via median sternotomy. Aortic cross clamping and cold cardioplegic liquid was applied for myocardial protection after initiation of hypothermic cardiopulmonary bypass. Single patch closure with Dacron pericardial patch or bovine pericardial patch was used in 19 cases (70.3%), following a technique similar to a famous study [12]. Eight cases were repaired by direct suturing without use of the patch. The ventriculotomy was closed by direct sutures. Concomitant CABG was performed in 16 patients (59.2%).

Paradoxically patients in the non-survivor group tended to be younger with a lower BMI. Both groups were equally distributed in the incidence of diabetes, hypertension, smoking, and dyslipidemia. There was high mean arterial pressure (MAP) and low heart rate (HR) in the survival group (95.39 vs. 73.33, P = 0.007, and 73.33 vs. 150.78, P = 0.043).

The majority of patients in the survival group received a form of early revascularization (83.3%), either percutaneous coronary intervention or thrombolysis. Delayed revascularization was associated with increased mortality (OR 17.500, 95% CI 2.365–129.506, P = 0.005). Logistic regression analysis demonstrated EF, three-vessel disease, Killip class, early surgery, and prolonged ionotropic support as predictors for mortality. Although not statistically significant, the use of post-operative MCS was less in the survivor group (9.61 vs. 25.78, P = 0.297) and four patients needed an upgrade to ECMO or LVAD. Interventions and complications are shown in Table 2 and logistic regression to analyze factors associated with mortality are summarized in Table 3. Patient profiles are summarized in Table 4.

**Table 2:** Interventions and complications between survival groups.

Interventions/Complications	Survivor (n = 18)	Non-survivors (n = 9)	P-value
**MCS**			
** IABP**	7 (38.9)	4 (44.4)	0.782
** ECMO**	12 (66.7)	6 (33.3)	0.099
** IABP + ECMO**	2 (11.1)	1 (11.1)	1
** LVAD**	2 (11.1)	3 (33.3)	0.161
**Change of MCS**	3 (16.7)	1 (11.1)	0.702
**Post-op days with MCS**	9.61 ± 4.44	25.78 ± 10.56	0.297
**Ionotropic support**	10 (55.6)	9 (100)	0.017
**Device to closure (Days)**	20.89 ± 7.09	19.78 ± 3.34	0.457
**Device thrombosis**	0	1 (11.1)	0.150
**Infection**	2 (11.1)	1 (11.1)	1
**Thromboembolic phenomenon**	1 (5.6)	1 (11.1)	0.603
**Revascularization**	15 (83.3)	2 (22.2)	0.002
**CABG**	11 (61.1%)	5 (55.5%)	0.004

Intra-aortic balloon pump (IABP); Extracorporeal membrane oxygenation (ECMO); Left ventricular assist device (LVAD); Mechanical support device (MCS).

**Table 3:** Clinical factors associated with mortality by logistic regression analysis.

Risk factors	B	SE	OR	95% CI	P-value
**EF**	0.279	0.116	0.756	23.283–30.050	0.016
**Three-vessel disease**	-4.085	1.304	0.017	0.001–0.217	0.002
**Killip Class**	2.531	1.166	12.571	1.280–123.480	0.030
**Early surgery**	-0.180	0.088	0.835	16.163–21.541	0.041
**Prolonged ionotropic support**	-0.371	0.149	0.556	0.368–0.840	0.013
**Delayed revascularization**	-2.862	1.021	17.500	2.365–129.506	0.005

Ejection fraction (EF).

**Table 4:** Patient profile.

Patient	Age (years)	Sex	Presenting duration of AMI (hours)	VSR diagnosis to surgery (days)	MCS duration to surgery (days)	Post-operative complications	Upgrade of MCS	Device complications (day)	Location of VSR	MCS duration after surgery (days)	ITC stay (days)	Hospital stay (days)	Outcome
**1**	68	M	25	21	18	None	No	None (NA)	Apical	1	5	27	Alive
**2**	49	F	46	26	21	None	No	None (NA)	Apical	1	6	23	Alive
**3**	62	M	71	15	11	None	No	None (NA)	Apical	2	5	13	Alive
**4**	70	M	96	14	12	None	No	None (NA)	Apical	1	4	36	Alive
**5**	75	M	16	14	11	ARF requiring RRT	No	None (NA)	Basal	1	5	95	Alive
**6**	63	F	42	17	11	None	No	None (NA)	Basal	2	5	12	Alive
**7**	59	M	25	25	22	None	No	None (NA)	Apical	2	4	24	Alive
**8**	70	M	27	34	17	None	No	Infection (11)	Apical	2	5	19	Alive
**9**	68	M	54	12	9	None	Yes	None (NA)	Apical	1	6	64	Alive
**10**	83	M	43	11	7	Re-exploration of bleeding	Yes	None(NA)	Basal	1	6	12	Alive
**11**	76	F	23	24	7	None	No	Infection (6), thromboembolic phenomenon (7)	Apical	2	7	16	Alive
**12**	65	M	51	28	22	Re-exploration of bleeding	No	None (NA)	Apical	2	7	15	Alive
**13**	58	M	26	21	16	None	No	None (NA)	Basal	3	7	24	Alive
**14**	78	M	13	25	14	None	No	None (NA)	Basal	1	6	19	Alive
**15**	67	M	56	23	10	None	Yes	None (NA)	Apical	1	5	26	Alive
**16**	56	M	22	25	20	ARF not requiring RRT	No	None (NA)	Apical	2	4	31	Alive
**17**	55	M	19	10	9	None	No	None (NA)	Apical	3	3	28	Alive
**18**	61	M	21	31	21	None	No	None (NA)	Apical	1	6	11	Alive
**19**	56	M	56	14	11	None	No	Infection (7)	Apical	3	9	38	Dead
**20**	82	F	32	23	20	ARF requiring RRT, DIC	No	None (NA)	Apical	1	11	43	Dead
**21**	61	F	23	17	8	DIC	No	Infection (8)	Apical	2	12	28	Dead
**22**	53	M	19	17	8	ARF not requiring RRT	No	None (NA)	Basal	2	14	40	Dead
**23**	59	M	68	12	12	None	Yes	None (NA)	Basal	1	10	109	Dead
**24**	65	F	14	15	12	None	No	Device thrombosis (2)	Basal	2	8	83	Dead
**25**	71	F	41	10	10	DIC	No	None (NA)	Apical	3	19	43	Dead
**26**	61	M	78	11	8	Re-exploration of bleeding	No	None (NA)	Basal	1	17	35	Dead
**27**	63	M	43	14	11	None	No	Infection (4)	Apical	2	16	111	Dead

The overall mortality after one-year was 33% with surgical mortality of 11%. Fig 1 shows a Kaplan Meier survival curve with a cumulative one-year survival of 66%. Complications related to ECMO and LVAD occurred in four patients. There were three inguinal infections and a device thrombosis in non-survivor group and two infections and one thromboembolic phenomenon in survivor group.

**Fig 1:** Kaplan Meier curve showing survival after one year.

## Discussion

Our study validates preceding observations that delayed VSR repair, undergone after 10 days of diagnosis was associated with a significant survival benefit. However, MCS did not show a statistically significant survival benefit. Prolonged use of inotropes conferred a higher risk of death. Similarly, three-vessel disease and higher Killip class were associated with an increased risk of mortality. There was no survival benefit from reperfusion. Although, early presentation to emergency, single-vessel disease, high mean arterial pressure (MAP), and heart rate (HR) were associated with better survival.

Non-survivors had more percentage of three-vessel disease (77.8% vs. 5.6%, p = 0.001), higher duration of MI to hospital presentation (41.56 ± 22.19 vs. 37.56 ± 21.89, p = 0.007), and a decreased MAP (73.33 ± 3.50 vs. 95.39 ± 5.81, p = 0.007). A left heart catheterization was performed on all the patients and delayed revascularization was associated with increased mortality. This is in contrast to a case-series that analyzed 14 patients retrospectively. It demonstrated no survival benefit in patients with revascularization. In addition, PCI was found only in the non-survivors indicating an increased mortality association [13]. Our study confirms better survival with early reperfusion, supporting the results of GUSTO-I and GRACE trials [14, 15]. However, patients undergoing PCI had higher mortality in both the SHOCK and APEX-AMI trials [16, 17]. This infers a heterogeneous result in our study and present literature.

MCS were used in all the patients in our study. While there was no statistically significant association with survival, a shorter duration of MCS was seen in the survivor group postoperatively. Data on MCS is mostly limited to IABP in case reports and case-series which show an improved survival after surgical repair [18]. However, in a retrospective study of 2,876 patients, the use of IABP increased all-cause mortality [8]. The data on ECMO is also limited to case reports and no significant studies have been done in evaluating the mortality benefits in VSR with cardiogenic shock. Our results show no statistical significance of MCS use in overall survival. The main benefit is in the hemodynamic support until surgical repair is feasible.

All the patients underwent VSR repair with or without concomitant CABG. Surgical timing ranged from 10 to 34 days. According to the American College of Cardiology/American Heart Association (ACC/AHA), emergent VSR repair is required regardless of the hemodynamic status [19]. We observed that deferred surgical repair was associated with an increased survival benefit. The overall mortality from our study was 33.3% which is lower than The Society of Thoracic Surgeons Adult Cardiac Surgery Database (STS-ACSD) study which was 42.9% [8]. One of the advantages of our strategy is hemodynamic stabilization before surgery, which confers a low operative risk and a favorable outcome. Another possible advantage is the healing of the infarcted myocardium leading to scar tissue formation. This fibrous myocardium enables stable repair and sutures. The healing process of the infarcted myocardium starts as early as the seventh day after MI. It takes 3–5 weeks more for a complete scar construct [20]. Thus, the idea of deferred surgical repair is to get an adequate scar formation. Our average duration of VSR diagnosis to surgical repair was approximately 20 days in both survival groups. Early surgery was associated with increased mortality in our study.

One disadvantage of prolonged deferral is the complications associated with MCS. One study reports major bleeding in 71.4% of patients on ECMO before VSR repair. They reported infection in all the cases [21, 22]. Unlike this study, their average duration of ECMO use was 12 days. We observed a lower rate of infection with only 11.1% of cumulative infection rate and one thrombosis of LVAD in a non-surviving patient. This contradicts previous studies that demonstrate increased complications with ECMO as the duration of days extends. Therefore, we believe that delayed surgery can be performed safely with MCS.

There are a few limitations of this study. First, the small sample size resulted in inadequate statistical power despite differences in the survival groups. The follow-up was adequate but the retrospective nature of the study limits the control of confounding factors. Surgical techniques were variable based on the expertise of the performing surgeon. Clinical and technical decisions for MCS were not controlled and were based on clinical judgment.

## Conclusion

Preoperative MCS and deferred surgery can improve survival in patients with post-MI VSR complicated by cardiogenic shock. Delayed reperfusion had an associated increased all-cause mortality. The key to better survival seems to be hemodynamic stabilization rather than MCS. This requires further investigation, specifically the optimal duration of support.

## Supporting information

S1 File Supporting file is available with the manuscript. (SAV)
